The article "Comprehensive assessment of cavernosography with 320-row dynamic volume CT versus conventional cavernosography in erectile dysfunction patients caused by venous leakage" was published in 2017. Journal: Biosci Rep.

# Comprehensive assessment of cavernosography with 320-row dynamic volume CT versus conventional cavernosography in erectile dysfunction patients caused by venous leakage

**DOI:** 10.1042/BSR20170112

**Published:** 2017-05-11

**Authors:** Cheng-Cheng Xu, Yu-Ning Pan, Yi-Fan Tang, Jie Zhang, Guo-Yao Wang, Qiu-Li Huang

**Affiliations:** 1 Department of Imaging, Ningbo First Hospital, Ningbo 315010, P.R. China; 2 Department of Urology, Ningbo First Hospital, Ningbo 315010, P.R. China

**Keywords:** 320-row DVCT cavernosography, Conventional cavernosography, Diagnostic and prognostic value, Erectile dysfunction, Venous leakage

## Abstract

The present study aims to investigate and compare the diagnostic and prognostic value of cavernosography with 320-row dynamic volume computed tomography (DVCT) versus conventional cavernosography in men with erectile dysfunction (ED) caused by venous leakage. A total of 174 patients diagnosed with ED were enrolled and received cavernosography with 320-row DVCT (DVCT group) and conventional cavernosography scans (control group) respectively. The diagnosis, complications, and prognosis of patients were evaluated. The DVCT group provided high-resolution images with less processing and testing time, as well as lowered radiological agent and contrast agent compared with the control group. In the DVCT group, 89 patients who were diagnosed with venous ED had six various venous leakage, namely superficial venous leakage, profundus venous leakage, the mixed type, cavernosal venous leakage, crural venous leakage, and also venous leakage between the penis and urethra cavernosum (9, 21, 32, 6, 18, and 3 cases respectively). Similarly, 74 patients out of the 81 who suffered from venous ED were classified to have superficial venous leakage (11), profundus venous leakage (14), the mixed type venous leakage (26), and middle venous leakage (23). Six out of 25 patients in the DVCT group, had improvements in ED while the remaining 19 achieved full erectile function recovery with no penile fibrosis and erectile pain. Cavernosography with 320-row DVCT is a reliable system that can be used to diagnose ED caused by venous leakage. This is especially useful in accurately determining the type of venous and allows for a better prognosis and direction of treatment.

## Introduction

Erectile dysfunction (ED) is been defined as the recurrent or consistent inability to generate or maintain a penile erection of sufficient rigidity for sexual intercourse [1]. It is a prevalent medical condition that affects the life quality in all male age groups. Current statistics show that it has affected 152 million males in 1995 and is projected to affect 322 million males globally by the year2025 [2]. Aging is one main risk factor contributing to the onset of ED, whereby data show a 20–40% occurrence rate in men aged between 60 and 90 years old and 50–100% in men who are between 70 and 80 years old [3]. Other risk factors such as depression, diabetes, heart disease, hypertension, atherosclerosis, high cholesterol, high blood pressure, obesity, and alcoholism are also in tight association with ED incidence, whereby vascular disease is found to be the highest contributing factor [4]. Causes of vasculogenic ED include arterial insufficiency (AI, 30%), mixed vascular etiology (10%), and veno-occlusive dysfunction (VOD, 15%), and VOD is a condition that occurs due to an inability to trap blood in the tunica albuginea of the corpora, which results in insufficient compression of the subtunical venules in the phase of full erection [5].

VOD, previously known as venous insufficiency or venous leakage, is a common occurrence of ED patients as well as patients who suffer from ED caused by penile arterial incompetence [6]. Cavernosography or cavernosometry has been adapted to evaluate VOD among male patients with a proposed organic ED [7]. Since the 1970s corpus cavernosography of the penis has been used to help elucidate the penile venous anatomy [8]. However, conventional cavernosography does not always reveal precise penile veins of interest due to overlapping by other veins, bone, or cavernous body. The obstruction of visualization of these structures also makes it difficult to show the origin of the veins through radioscopy [9]. With new advancements made in medical imaging technology, like computed tomography (CT) and also magnetic resonance imaging (MRI), more knowledge and information about the corpus cavernosum has been obtained [10]. Currently, improvements in the CT scan from 64 to 320 slice provide us with a higher resolution and much more detailed structure images, allowing for superior visualization of the internal penile tissue [11]. Furthermore a current diagnostic tool, dynamic volume computed tomography (DVCT), is characterized by 320 slice detectors with 350 ms gantry rotation, a 5 mm thickness as well as a wide coverage range of 16 cm in the *z*-axis, and it can cover the whole heart within one cardiac cycle [12]. Hence, our purpose of the present study is to comprehensively assess DVCT cavernosography and conventional cavernosography for men with ED caused by venous leakage.

## Materials and methods

### Ethical statement

The present study was approved by the Ethics Committee of the Medical Faculty of Ningbo First Hospital. The written informed consents were obtained from all patients or their families.

### Study subjects

From June 2014 to June 2015, 174 patients diagnosed with ED in Ningbo First Hospital were recruited in our study, among which 93 patients received DVCT cavernosography and 81 patients received conventional cavernosography. The inclusion criteria were as follows: (1) patients who were preliminarily confirmed with ED by detailed inquiry of disease history, physical examination, and laboratory tests before grouping; (2) patients who showed no erection or ED three audio visual sexual stimulations (AVSS) and nocturnal penile tumescence; (3) velocity of cavernosal artery was measured by duplex ultrasonography prior to admission. The exclusion criteria included: (1) patients who suffered from psychogenic ED, neurogenic ED, and endocrine ED; (2) those who suffer from disease- and drug-induced ED; (3) external arterial ED; (4) allergies to contrast medium; (5) patients who suffered from liver and chronic kidney dysfunction.

### Detection of blood biochemical indices

A week before undergoing cavernosography, the blood biochemical indices of patients were detected on an empty stomach in the morning. These biochemical indices include: hemoglobin A1c (HbA1c), fasting plasma glucose (FPG), total cholesterol (TC), triglyceride (TG), high-density lipoprotein (HDL), and low-density lipoprotein (LDL).

### Cavernosography with 320-row DVCT

An iodine allergy test was performed for all patient with a vein needle dwelling the same day on one upper limb before being scanned by a 320-row DVCT. Patients were told to lie down, while the nurses completed the intravenous infusion and connected the CT scanner. The patients’ perineal positions were sterilized with 2% povidone-iodine and followed by injection of 30 mg of papaverine using a 5-gauge scalp needle in the middle of corpora cavernosum. This was done to induce an erection with a 3–5 min of compression on the puncture point. After 5 min, papaverine was increased to 60 mg for the patients who were not satisfied with their erection conditions. The venous accesses were unblocked immediately after the full erection was observed. Patients were injected with 80 ml iobitridol (350 mg/ml, Aulnay-sous-Bois) at the speed of 5 ml/sec mixed with 20 ml of normal saline for washing. During the full erection, cavernosography with 320-row DVCT was performed for four times at 2 s intervals during the arterial phase. After sterilization of the puncture point, diluted iohexol (ratio of 1:1, 20–60 ml) was injected into the erect cavernosa at the speed of 2–4 ml/sec using a 7-gauge scalp needle to obtain another erection. At the same time, cavernosography with a 320-row DVCT (Aquilion One, Toshiba America Medical Systems, CA, U.S.A.) was performed under the same conditions. The scanning parameters were set up as follows: field of view, 160 mm; slice thickness, 0.5 mm; scan speed, 0.75 s/rot; voltage of scanning tube, 80 kV; tube current, 150–310 mA.

### Image processing with 4D digital subtraction angiography

A total of 3200 images with 0.5 mm slice thickness were produced in each scan (each volumetric data containing 320 images). Computer software 4D-digital subtraction angiography (4D-DSA; Toshiba Corporation, Tokyo, Japan) was used to reconstruct dynamic 3D angiograph. High-resolution images of lesion were obtained by means of pseudo color, rotation at any angle, local amplification, shielding, and other techniques.

### Conventional cavernosography examination

An iodine allergy test was performed before each cavernosography performed on the patient. Patients were first asked to lie in a dorsal decubitus position, and have their intestines and stomach checked and their perineal positions were sterilized and paved with sterile sheet. Penile prosthesis (0.2 ml) containing papaverine, phentolamine, and prostaglandin E was injected into the corpora cavernosa, with local compression for 1–2 min. An elastic band was initially ligated at the penile base followed by a manipulation of the penis to distribute the dosage uniformly around entire length of the corpora cavernosa in order to achieve and maintain full erection. A 9-Gauge needle containing 30% meglumine diatrizoate (30–60 ml) was injected at the rate of 30 ml/min into the penile base at 45 degrees oblique, 0.8 cm below the coronary sulcus of the corpora cavernosa. Conventional cavernosography was performed at 30, 60, 90, 120, and 900 s respectively, after the contrast medium was injected. Upon caversonaography completion, needles were pulled out and compression was performed for 1–2 min. Observation and data recording lasted for at least 5 min, during which leakage of contrast medium and hematoma should be prevented.

### Statistical analysis

SPSS 21.0 software (SPSS, Inc, Chicago, IL, U.S.A.) was used for statistical analysis. The count data were expressed as a percentage. An *X*^2^ test was used to compare data between different groups. Measurement data were displayed as mean ± standard deviation. For a comparison between two groups, independent sample *t* test was performed. Values of *P*<0.05 were considered as statistically significant. The whole experiment was repeated three times under the same condition in order to obtain an average value.

## Results

### Baseline characteristics of patients between the DVCT and control groups

In this investigation, 81 patients (age between 21 and 59 years old with a mean age of 29.40 ± 2.10 years and duration of ED ranging from 7 months to 11 years) received conventional cavernosography and 93 patients (age between 19 and 56 years old with a mean age of 29.70 ± 2.30 years and ED course ranging from 6 months to 8 years) received cavernosography with 320-row DVCT. There were no significant differences in age, course of disease, and history of marriage, smoking and drinking between the two groups (all *P* >0.05) (Table 1).

**Table 1:** Comparisons of baseline characteristic between the DVCT and control groups

Characteristic	Control group (*n*=81)	DVCT group (*n*=93)	*t*/*χ*^2^	*P*
Mean age (years)	29.40 ± 2.10	29.70 ± 2.30	0.894	0.373
Course of disease	5.7 ± 1.2	5.4 ± 1.3	1.573	0.117
Marriage history (Y/N)	45/36	58/35	0.754	0.362
Smoking history (Y/N)	43/38	52/41	0.892	0.709
Drinking history (Y/N)	59/22	66/27	1.097	0.784
Hypertension (Y/N)	42/39	40/53	1.427	0.244
HbA1c (%)	7.62 ± 1.42	7.55 ± 1.35	0.333	0.740
FPG (mmol/l)	8.61 ± 0.23	8.71 ± 0.51	1.626	0.106
TC (mmol/l)	4.85 ± 0.64	5.01 ± 0.78	1.466	0.145
TG (mmol/l)	1.80 ± 0.29	1.87 ± 0.30	1.559	0.121
HDL (mmol/l)	1.13 ± 0.21	1.21 ± 0.36	1.756	0.081
LDL (mmol/l)	2.57 ± 0.33	2.66 ± 0.45	1.485	0.139

Note:Y, yes; N, no.

### Comparison of the basic features of cavernosography with 320-row DVCT and conventional cavernosography

Compared with control groups, the DVCT group provided high-resolution images with less time for processing and type of detection, as well as lesser doses of radiological agent and contrast agent administrated to the patients (all *P*<0.05), as shown in the Table 2.

**Table 2:** Comparison of general features of cavernosography with 320-row DVCT and conventional cavernosography

Feature	Conventional group (*n*=81)	DVCT group (*n*=93)	*t*/*χ*^2^	*P*
Image processing time (min)	7.6 ± 2.1	3.7 ± 1.2	12.810	*<* 0.001
Radiation dose (mSv)	6.5 ± 1.4	4.5 ± 1.1	9.486	*<* 0.001
Testing time (s)	577 ± 148	481 ± 156	4.147	*<* 0.001
Contrast dose (ml)	80.6 ± 11.5	66.5 ± 10.1	11.570	*<* 0.001

Note: DVCT cavernosography, cavernosography with 320-row dynamic volume CT.

### Images for typical features of ED in the DVCT and control groups

Images produced by cavernosography with 320-row DVCT show smooth, symmetrical, high-density spindle-shaped corpora cavernosa, and strip-like low-density shadows in the space of corpora cavernosa in the DVCT group (Figure 1A and B). This is a visual confirmation the 93 patients were indeed suffering from ED. Images produced by conventional cavernosography show symmetrical smooth-edge, high-density images in corpora cavernosa, and strip-like low-density shadows in the interval of corpora cavernosa were observed in the control group (Figure 1C and D). This is also a confirmatory sign that these 81 patients also suffer from ED.

**Figure 1:** Image of corpora cavernosum detected by the cavernosography with 320-row DVCT compared with an image taken by conventional cavernosography (**A**) Cavernosography with 320-row DVCT image of regular cavernosa by; (**B**) cavernosography with 320-row DVCT image of cavernosal venous leakage by; (**C**) conventional cavernosonography image taken of the regular cavernosa by; (**D**) conventional cavernosa image of the cavernosal venous leakage by DVCT.

### Venous leakage of corpora cavernosa in patients scanned by cavernosography with 320-row DVCT

Cavernosography with 320-row DVCT displays no venous drainage in four out of the 93 patients, indicating that these cases were of non-venous ED etiology. The rest of the patients showed different venous leakages, including nine cases (10.1%) of superficial venous leakage (Figure 2A). These patients exhibited abnormal structures of the superficial dorsal penile vein that traced all the way to the superficial external pudendal vein, superficial femoral vein, and other branches of the great saphenous vein. We found 21 cases (23.6%) of a profundus venous leakage etiology (Figure 2B), among them superficial dorsal veins were displayed with DVCT cavernosography dynamically tracing to the prostatic venous plexus, bladder venous plexus, and internal iliac vein, which all belong to common types of single venous leakages. Eighteen patients (20.2%) presented with crural venous leakage (Figure 2C), whereby their penile veins were abnormally displayed that flowed into the internal jugular vein; six patients (6.7%) of cavernosal venous leakage (Figure 2D); three patients (3.4%) of venous leakage between the penis and urethra cavernosum (Figure 2E), which is the rare type; the remaining 32 patients (36.0%) were of mixed venous leakage, among them a mix of more than two kinds of venous leakages were detected (Figure 2F).

**Figure 2:** Venous leakage of corpora cavernosa scanned by cavernosography with 320-row DVCT (**A**) Superficial venous leakage; (**B**) profundus venous leakage; (**C**) crural venous leakage; (**D**) cavernosal venous leakage; (**E**) venous leakage between the penis and urethra cavernosum; (**F**) mixed venous leakage.

### Venous leakage of corpora cavernosa scanned by conventional cavernosography

Conventional cavernosography showed no cavernous bodies in seven patients, suggesting that ED were caused by psychogenic ED. Based on the X-ray findings, venous ED was classified into four types. Eleven patients (14.9%) were classified in type I—superficial venous leakage. This type of venous leakage is classified by the development of external jugular veins, the great saphenous vein, femoral vein, and external iliac vein were observed (Figure 3A). Twenty three (31.1%) exhibited type II—middle venous leakage, among them developed corpora spongiosum, glans penis (Figure 3B), prostatic venous plexus, prostatic venous plexus, inferior vena cava, internal iliac vein (Figure 3C), and deep dorsal vein of penis. Cavernosa was slightly exposed, accompanied by corpora spongiosum and deep dorsal vein of penis in type II middle venous leakage. A total of 14 (18.9%) were of type III—profundal venous leakage, in which development of deep veins of penis and internal jugular veins were observed (Figure 3D). The remaining 26 patients (35.1%) belonged to type IV—mixed leakage, which was demonstrated as two or three characteristics of the images of type I, II, and III (Figure 3E and F).

**Figure 3:** Venous leakage of corpora cavernosa scanned by conventional cavernosography (**A**) Type I: superficial venous leakage (imaging of left external iliac vein); (**B**) Type II: middle venous leakage (imaging of corpora cavernosum urethrae and glans penis); (**C**) Type II: middle venous leakage (imaging of right internal iliac vein); (**D**) Type III: profundus venous leakage (imaging of deep veins of penis and internal jugular vein); (**E**) Type IV: mixed leakage (imaging of left internal iliac vein, deep veins of penis, and internal jugular vein); (**F**) Type IV: mixed leakage (imaging of left internal iliac vein, glans penis, deep veins of penis, and internal jugular vein).

### Comparison of adverse reactions of patients in the DVCT and control groups

Cavernosography with 320-row DVCT scans, the DVCT group had shown that three cases suffered from symptoms of dizziness, palpitation, sweating, and hot flushes after injection of papaverine (30 mg). However, these symptoms were disappeared and rested for after 5 min. In contrast, eight cases showed priapism, which was relieved by drainage of cavernous sinus whereas 23 cases exhibited penile subcutaneous congestion. In the control group, we recorded five cases of foreskin hematoma, three cases of contrast agent leakage to the skin, and five cases with the side effects after vasoactive drugs. Symptoms after vasoactive drug administration included three cases of dizziness and palpitation and two cases of priapism. All of the adverse reactions produced were dealt with by proper treatment. Our results showed that there was significant difference in the penile subcutaneous congestion and foreskin hematoma between the DVCT and control groups (*P*<0.05), which might be resulted from loose or short-time local compression. No other significant differences in other adverse reactions were detected between the two groups (*P*>0.05), as demonstrated in the Table 3.

**Table 3:** Comparison of the rate of adverse reactions between the DVCT and control groups

Adverse reactions	Control group (*n*=81)	DVCT group (*n*=93)	*t*/*χ*2	*P*
Dizziness, palpitation, sweating, and hot flushes	3	3	1.154	0.863
Priapism	2	8	0.27	0.083
Penile subcutaneous congestion	0	23	0.018	<0.001
Foreskin hematoma	5	0	13.44	0.015
Contrast agent leakage to the skin	3	0	8.338	0.061

### Result of penile operations after cavernosography with 320-row DVCT and conventional cavernosography

In the DVCT group, 31 patients with venous leakage received various operations and surgical procedures. These procedures included ligations of deep dorsal penile vein (6 patients), embedding of deep dorsal penile vein and crural vein ligations (12 patients), and ligations of penile crural vein (13 patients). In the control group, 15 ED underwent operations including ligations of deep dorsal penile vein (3 patients), embedding of deep dorsal penile vein and crural vein ligation (7 patients), and penile crural vein ligations (5 patients), as revealed in the Table 4.

**Table 4:** Operations after cavernosography with 320-row DVCT and conventional cavernosography

Surgical treatment	Control group (*n*=81)	DVCT group (*n*=93)
Surgical treatment	15 (18.52%)	31 (33.33%)
Ligations of deep dorsal penile vein	3 (3.70%)	6 (6.45%)
Embedding of deep dorsal penile vein and crural vein ligations	7 (8.64%)	12 (12.90%)
ligations of penile crural vein	5 (6.17%)	13 (13.98%)

### Follow-up

In the DVCT group, 25 out of 31 cases received follow-up studies. Among these patients, 6 of them showed improvements in erection whereas 19 patients fully recovered from ED. Patients, who received operations, were treated with either phosphodiesterase 5 inhibitor (PDE5) or vacuum negative pressure pump therapy according to their own choice and disease severity. Some patients additionally conducted cavernosography with 320-row DVCT to evaluate their current disabilities. Positive observation was implemented according to each patient’s will. In the postoperative follow-up of patients in the control group, no penile fibrosis or erectile pain was observed.

## Discussion

ED is a chronic disorder that is increasingly prevalent with age in males [13]. It is defined as the inability to attain and maintain an erection during satisfactory sexual intercourse. Various etiological factors attributing to ED include hormonal, psychological, arterial, neurologic, or cavernosal impairment [14]. In the present study, we utilized the newly developed cavernosography with 320-row DVCT to compare findings with those obtained by conventional cavernosography. We do this to comprehensively assess both of the cavernosography as tools to help diagnose venous ED. Our findings revealed that DVCT cavernosography is promising diagnostic tool in the diagnosis of patients with venous ED.

In the present study, 89 out of 93 patients in the DVCT suffered from venous leakages at various sites, which we could clearly detect. We also found five types of venous leakages in 74 out of the 81 patients in the control group. One study revealed that three-dimensional (3D) CT cavernosography provides high-resolution images for the venous drainage from any angle and clearly shows anatomical structures such as drainage veins, including dorsal veins, cavernous veins, crural veins as well as other emissary veins [9]. Moreover, a novel venous leakage classification using multi-detector (MDCT) cavernography revealed the leakage commonly seen in the deep dorsal vein and superficial vein [15]. Chen et al. introduced ultrasonography as a method of assessment for vasculogenic impotence in 1985 and prior studies has proved ultrasound a major tool applied in the vascular differentiation process in ED [16,17]. In addition to ultrasounds, cavernosography has also been used by urologists to produce some of the earliest images taken of erect corpus cavernosum [10]. However, most venous vasculatures are covered in penile venous distribution when observed under ultrasonography, while conventional pharmaco-cavernosography only reveals a small portion of the leaky deep dorsal vein and fails to display either the para-arterial veins (PAVs) or the cavernosal veins (CVs) [8]. Dynamic infusion cavernosometry or cavernosography was used to diagnose corporal veno-occlusive dysfunction (CVOD) in a study performed on aged rats, but it failed to reveal the histological changes related to CVOD, including an increase in corporal fibrosis and a decrease in corporal smooth muscle cells [18]. A comparative study prospectively studied the accuracy and radiation dose of invasive coronary angiography (ICA) and DVCT for the coronary artery disease (CAD), with the result showed the effective radiation dose by DVCT declined significantly than that of ICA [12] A detection of CADs scanned by a 320-detector row DVCT demonstrated that DVCT produced detailed images and high accuracy [12]. Besides, the application of multi-segment reconstruction can be more feasible with the DVCT employment [19]. Thus, we reached a conclusion that cavernosography with 320-row DVCT might be an alternative method for DVCT detection as it provides more information regarding various venous leak and subtypes in accordance with the studies above.

Considerable differences were seen in the diagnosis of venous leak sites between the control and DVCT groups. The DVCT group provided us with high-resolution images with less processing time, as well as required lesser doses of radiological and contrast agent compared with the control group. CT perfusion imaging along with the rest and adenosine stress 320-row CT is identified as an accurate method in detecting myocardial ischemia caused by obstructive atherosclerosis as compared with single photon emission computed tomography (SPECT) [20]. George et al. used the large area coverage of the 320-detector row scanner to conduct a triple rule-out protocol in 30 patients, which hold the promise in conducting a rapid high quality ‘triple rule-out’ test with no high contrast load, four-dimensional CT subtraction angiography and enhanced myocardial perfusion imaging comparing with those when the conventional scans were used [21]. Another study revealed that the effective dose was reduced as much as 91% in volume scanning relative to conventional scanning [22]. The 320-detector row scanner is equipped with a standard temporal resolution of nearly 175 ms, which is 50% shorter than the gantry rotation time, and it remains longer than 33 ms of catheter coronary angiography operating at speed of 30 frames/s, aiming to achieve images of excellent quality [21]. The result of a previous study of scans on the coronary arteries also showed that a 320-detector row scanner developed high-resolution images in almost 90% of coronary artery segments with low heart rates were reduced [19]. This is very useful in clinical settings to help diagnose and treat patients.

Our investigation showed that the cavernosography with 320-row DVCT is a promising tool in clinical application. However, there are some problems concerning in cavernosography with 320-row DVCT compared with conventional one or MRI, including the radiation exposed to patient, movement of the bed in the process of scanning, and difficulty in examining the patient [9]. Our study is among the few that evaluates the diagnostic abilities between the cavernosography with 320-row DVCT and conventional cavernosography. We hope that it provides further evidence in the advantages of DVCT cavernosography for examining ED in patients pertaining to venous leakage etiology.

## Abbreviations

4D-DSA: 4D-digital subtraction angiography
AI: arterial insufficiency
AVSS: audio visual sexual stimulations
CAD: coronary artery disease
CT: computed tomography
CV: cavernosal vein
CVOD: corporal veno-occlusive dysfunction
DVCT: dynamic volume computed tomography
ED: erectile dysfunction
FPG: fasting plasma glucose
HbA1c: hemoglobin A1c
HDL: high-density lipoprotein
ICA: invasive coronary angiography
LDL: low-density lipoprotein
MRI: magnetic resonance imaging
PAV: para-arterial vein
PDE5: phosphodiesterase 5 inhibitor
SPECT: single photon emission computed tomography
TC: total cholesterol
TG: triglyceride
VOD: veno-occlusive dysfunction
